RETRACTED

# Visual Information Features and Machine Learning for Wushu Arts Tracking

**DOI:** 10.1155/2021/6713062

**Published:** 2021-08-04

**Authors:** Jing Li, Guangren Zhou

**Affiliations:** ^1^Sports Center, Xi'an Jiaotong University, Shaanxi 710049, Xi'an, China; ^2^School of Comprehensive Foundation, Wannan Medical College, Wuhu 241002, Anhui, China

## Abstract

Martial arts tracking is an important research topic in computer vision and artificial intelligence. It has extensive and vital applications in video monitoring, interactive animation and 3D simulation, motion capture, and advanced human-computer interaction. However, due to the change of martial arts' body posture, clothing variability, and light mixing, the appearance changes significantly. As a result, accurate posture tracking becomes a complicated problem. A solution to this complicated problem is studied in this paper. The proposed solution improves the accuracy of martial arts tracking by the image representation method of martial arts tracking. This method is based on the second-generation strip wave transform and applies it to the video martial arts tracking based on the machine learning method.

## 1. Introduction

The extraction of visual image information features is a crucial problem of computer vision and intelligent image processing. It is also an essential technology, which has received extensive attention in the past 20 years. It mainly refers to using a computer algorithm to extract the representative image information in the image to determine whether a point is a unique factor for identification. The standard image features can be divided into local features and global features from the representation range of their features. The content of image features can be divided into the corner, edge, contour, histogram, region, etc. Distinguishing particular features is the most fundamental basis of computer vision and image information understanding. Its basic meaning is generating a dimension vector that can reflect the essential characteristics of the recognized pattern according to the input system information. Therefore, the selection of features has become the most fundamental basis for computer judgment. The most crucial feature of feature extraction is “repeatability”: the features extracted from different images of the same scene should be the same, in which the computer can repeatedly select. For example, features make it possible to find similar martial arts structures in multiple motion images. These can be used as the model input for further selection and processing. In essence, the martial arts tracking method based on machine learning is to extract appropriate features and add appropriate machine learning algorithms. The quality of feature extraction can directly affect the classifier's performance and the final detection result [1, 2].

RETRACTED

The machine learning method can be divided into classification and regression according to the data category and discrete degree. Classification can be seen as finding a label that belongs to a particular class in a discrete category for given data. Generally, it can be described as follows: a training sample set is known, which is the feature set of a sample, and usually expressed in the form of a vector. Each element of the vector is a description of an inevitable feature of the sample and is a label of the sample's category. What we want to establish is a classification rule. For any unknown sample, we can apply this rule to its eigenvector to determine the sample category. Regression is to make accurate predictions or estimate the label's continuous real value corresponding to the data, which is the specific real value [3].

For continuous and comprehensive trend estimation in the real number space, the corresponding label in this problem is the continuous space, such as the posture coordinate value of three-dimensional joint points in each image of martial arts. The machine learning method of Wushu motion tracking is to estimate the value of the 3D posture corresponding to the image space. The standard models of discriminant tracking methods include parametric methods and nonparametric methods, such as NNK, Kr, local GP, shared Golem, and skill. The data association is shown in Figure 1, which is the low-dimensional popular or implicit variable space of data features [4].

However, generally speaking, many machine learning methods are derived from some basic ideas. The most typical and representative is the Gaussian process [5].

## 2. Machine Learning Methods in Wushu Arts

A Gaussian regression process is a set of random variables, and any numbers of its finite subsets are subject to the joint Gaussian distribution. The Gaussian process has been widely studied in martial arts tracking. It poses a recovery in recent years because of its output probability distribution, function continuity, and other characteristics. However, we do not know the spatial distribution characteristics of a specific sequence of martial arts postures. Any traditional data distribution (martial arts postures are no exception) is infinitely close to a Gaussian normal distribution under the massive statistical results. Learning the Gaussian process means learning the superparameters of the method instead of learning the weights of the primary functions often contained in traditional machine learning methods. A parameter edge process can eliminate the corresponding weight to reduce the extra parameters. In other words, the superparameters are learned through a maximum likelihood function. Here, the parameters are not the standard mean and variance matrix of traditional data statistics but the mean and variance functions. In other words, a Gaussian process is entirely determined by its mean function and covariance function. As long as the mean function *m*(*x*) and covariance function *k*(*x*, *x*′) are determined, the Gaussian process is entirely determined. In regression estimation, a kernel function is selected to assume the prior distribution of the data. A posterior part of the function is obtained by combining the primary and training data used to estimate the new data [6–8].

RETRACTED

The traditional machine learning methods are studied on the premise that the number of samples is enough. The performance of the proposed methods is theoretically guaranteed when the total number of samples tends to infinity when the number of samples is enough. However, in most practical cases, the number of samples is limited. Therefore, it is difficult to achieve the desired results. However, the Gaussian process finds a method to predict multiple repetitions through limited data. The predicted data space is nearly infinite. Therefore, GPR can be used to represent the nonlinear input-output mapping, such as martial arts tracking [9]. The machine learning problem can be expressed as there is a specific dependence between the known variable *y* and the input *x*. In other words, there is an unknown joint probability distribution *F*. The machine learning problem estimates the maximum posterior probability according to *n* different samples. GPR represents a Bayesian function with Gaussian distribution [10]. However, generally speaking, many machine learning methods are derived from some basic ideas. The most typical and representative is the Gaussian process.

(1) $$\begin{array}{c} p\left(f|X\right)=N\left(0,K\right), \end{array}$$

where *f*=[*f*_1_∧∧, *f*_*n*_] is a series of data spaces with function value and *f*_1_=*f*(*x*_1_) is the feature vector of the original image. *X*=[*X*_1_ … …*X*_*N*_]^*T*^ is a covariance matrix, and *K* is a covariance function *K*_*i*,*j*_=*k*(*x*_*i*_, *x*_*j*_). In the actual operation process, we have assumed that the data are Gaussian distribution. Hence, a radial basis function (RBF) or a Gaussian kernel function can be represented by the data association. For example, consider the function *K*_*R*_(*x*_*i*_, *x*_*j*_)=exp(−*γ*_*x*_‖*x*_*i*_−*x*_*j*_‖^2^)+*λ*_*x*_*δ*_*ij*_, where *γ*_*x*_=0 is the kernel width parameter. *λ*_*x*_=0 is the noise difference. *γ*_*x*_=0 is the Kronecker trigonometric function, if the value is 1, other cases are 0. Since the prior of the joint distribution is Gaussian distribution, the posterior prediction of the new data is based on the output value of the observed samples. The mean and variance are as follows:

(2) $$\begin{array}{c} m\left(y^{\left(d\right)}\right)=Y^{\left(d\right)}K_{x}^{-1}K_{x}^{s},\\ \sigma^{2}\left(y^{\left(d\right)}\right)=K_{x}\left(x,x\right)-{\left(K_{X}^{x}\right)}^{T}K_{X}^{-1}K_{X}^{x}. \end{array}$$

From the perspective of the graph structure, the Gaussian process can be recognized as a potential structural association between any observed data pair. The square node is the observed vector, and the circular node is the unobserved vector. Each sample pair obeys Gaussian distribution, and the data are also interrelated, which affects the estimation of other variable functions [11–13].

RETRACTED

Besides, any machine learning process similar to the Gaussian process involves the problem of data generalization or generalization ability. This is how we use the existing data to fit the data distribution of unknown results as much as possible and infer the existing observations into a more comprehensive problem space [14]. The generalization ability of the data is one of the basic requirements to test whether a machine learning algorithm has real wide availability. However, it is impossible to know precisely whether the test data are consistent with the sample space of the training data. According to the law of large numbers and the general situation of the whole data, most problems can be simplified as a Gaussian distribution or a linear superposition of multiple Gaussian distributions. The posterior distribution also conforms to the Gaussian theory. It can be believed that the Gaussian process reflects the complex correlation of the sample data to a certain extent [15]. The core of this correlation is the kernel function and covariance, which are mainly regulated by the parameters of the kernel function and some superparameters. Some parameters can be eliminated based on marginal parameters, but a superparameter itself needs further verification. Therefore, in GPR, the selection of parameters is a crucial problem. The parameters of different features need further cross-validation to avoid overfitting and underfitting [16–20].

## 3. Wushu Tracking Mechanism

The subject of Wushu tracking comes from the urgent research needs of computer vision in recent 20 years. As an essential branch of computer science and artificial intelligence, computer vision aims to use various electronic imaging systems to replace the human eye to obtain visual perception. The computer replaces the human brain to realize the processing and understanding of visual information [21–23]. In short, it is to make the computer have human visual recognition. A complete vision system usually involves the following contents: acquisition, processing, representation, storage, and transmission. First, the computer equipment based on control sensing collects the original data. Then, the acquired visual data are further characterized or compressed by the computer, analyzed, and processed. Then, the data are stored and transmitted through the network to realize a series of functions of human biological vision. Finally, the computer forms a clear and meaningful description of the collected image content to perceive the objective world visually. Visual information processing is the crucial and challenging point in the field of computer vision [24–27].

RETRACTED

### 3.1. Martial Arts Tracking Using the Second-Generation Band Wave Transform

The traditional representation method based on the image edge only describes the geometric characteristics of the image through the edge. It is not only not strict but also tricky to describe the image well, which hinders further effective feature representation and advanced computer vision processing. Therefore, Mallat introduced geometric flow to describe the geometric characteristics of images. Based on the first-generation bandelet, they proposed the second-generation strip wave transform. Based on the geometric flow of image characteristics, a new image feature extraction method in martial arts tracking based on the second-generation strip wave transform is proposed in this paper. This method extracts the top feature of geometric flow in the region direction, representing the main texture direction and change in the region direction. Because the representation of this method is sparse and scale-invariant, it can be used for illumination change. The main image also has good robustness (based on the change of the gray image level rather than brightness). It can distinguish the difference under the apparent deformation of the image. In this method, the statistical features of the bandelet in the bandelet transform are used as image features. The Gaussian and double Gaussian processes are combined to perform regression and track martial arts in the image [28, 29].

### 3.2. Geometric Flow Feature Extraction Method of the Strip Wave

The visual information of the image is the precondition of Wushu tracking. Using the geometric flow feature of the strip wave to extract the image features of martial arts can accurately express the movement posture and the general texture distribution in the image. As the most critical part of bandelet geometric flow feature extraction, our algorithm requires a full analysis of feature extraction early. The proposed algorithm uses the second-generation strip wave algorithm experiment to ensure that the specific feature extraction method [30–33] can extract the most suitable pattern and texture information of the characters in the image. The generated image [34] descriptor is unique and selective.

RETRACTED

### 3.3. Optimal Parameter Selection

When the bandelet transform is used for image compression, the primary purpose is to reduce the number of nonzero coefficients as far as possible. The parameters of the conventional bandelet transform are different from those of the martial arts tracking, which need to be determined by the parameter selection experiment. In terms of parameter selection, the experiment adopts the same method as 2, comparing the ROC curve after training the classifier with different transformation parameters to determine these parameters. Here, we choose the ROC curve of different detection rates for each possible false positive rate. The higher the ROC curve tends to the left vertex angle, the better the corresponding parameters are.

## 4. Results and Discussion

In this section, we described the results of the proposed scheme and explained them in detail.

### 4.1. Two-Dimensional Wavelet Transforms

We choose one to five layers of-dimensional wavelet transform and do not carry out two-dimensional wavelet transform, a total of six cases of experiments. Among them, *j* − max=2, *j* − min=2,and *T*=15, and the experimental results are consistent. When the wavelet level is 1-2, the ROC curve can present good detection results. Therefore, we choose an excellent wavelet transform. The obtained image features are used for tracking with good results, as shown in Figure 2.

The results obtained in this paper are consistent with those in the literature, and the best result is obtained by using only one layer of the two-dimensional wavelet transform. The main reasons are as follows: the more the decomposition level, the lower the representation ability of the feature of the higher layer's low-frequency approximation coefficient is compared to the better the high-frequency detail coefficient. Furthermore, using only one layer of the two-dimensional wavelet transform is also conducive to selecting the scale range of features in the process of tracking the predictor regression mapping, maintaining a unified quantization interval, and avoiding the instability caused by too extensive variation range of kernel parameters [35, 36].

### 4.2. The Scale of the Minimum Binary Partition and the Maximum Scale of Quadtree Upward

In theory, the smaller the minimum partition is, the larger *j* − min is and the more reasonable the quadtree *j* − max is. Larger *j* − max and smaller *j* − min will bring more time complexity to the process of feature extraction, which is not conducive to the learning of a vast database. The tracking error can be stabilized in a lower range, and the time required for feature extraction is significantly reduced to demonstrate that the average joint error of each frame of three-dimensional equine or human posture data on theoretical knot data is mm. Obviously, the lower the error, the more accurate the tracking. In the double Gaussian system with a neighbor pruning algorithm, the number of *k*-nearest neighbors is 100. As a result, a video sequence from the Humaniva database is selected for testing. When the 4 × 4 bandelet descriptor parameters are selected, the average joint error of each frame of the Wushu 3D pose data verified on the walking data is mm.

RETRACTED

It should be noted that the results of this group of experiments are consistent and generalizable. Suppose the same feature extraction method is used on similar motion data. The average effect of *j*-max = 2 and *j*-min = 2 will be better than that of other transform extraction features, and a 2-scale subdivision size is adopted. It can be seen that only 4 × 4 size blocks are used to extract features from the bandelet transform. A two-layer upward quadtree optimization merging strategy is adopted. It has the best representation ability and relatively low time consumption. At the same time, we further use the features of large and small blocks. Although the tracking effect will be slightly affected, it can significantly reduce the dimension of the descriptor.

### 4.3. Quantization Threshold *T*

The purpose of determining the quantization threshold *T* is to control the quantization range in the process of image signal quantization. The value whose coefficient is less than *t* is set to zero, thus omitting redundant information. In the image coding, *t* is used to control the compression ratio. The larger the value is, the higher the compression ratio is and the more pronounced the image distortion is. On the contrary, the selection of the quantization value affects the coefficient value more significantly than in a one-dimensional wavelet transform in a certain direction while searching for the optimal direction of geometric flow. Therefore, selecting too large or too small *t* is not conducive to finding the optimal direction of geometric flow. According to different application fields, the processing of the *T* value is also different. It is still necessary to find the best *t* value through specific experiments. When *Level* *=* *1, j*-max = 2, *j*-min = 2, and *T* = 15 are taken, good results are obtained. The small range variation of this value has no noticeable effect on the actual results. It can be seen from the existing literature and preliminary experiment 3 that the selection of *T* has little influence on the training error rate and test accuracy rate, which the diversity of photos should produce for the accurate extraction of martial arts image features.

RETRACTED

### 4.4. Block Size

For the influence of subblock size selection on the image signal, large or small subblock partition will have a deviation effect on the actual image feature extraction results. There is an optimal subblock size, and the subblock segmentation is too small or too large. We select 4 × 4 (or 8 × 8) subblock size for feature extraction and parameter selection in the actual experiment. This choice is mainly based on the size of the image and the dimension of the description features.

#### 4.4.1. Strip Wave Feature Extraction Using Algorithm Optimization

The implementation of the bandelet transform in the second generation of the bandelet transform involves a tedious sorting operation. We need to improve the algorithm further and reduce the sorting complexity of descriptor extraction. In the extraction process, the order of wavelet coefficients will be consistent for geometric flow blocks with the same scale and order. Therefore, the sorting index can be established in advance according to all possible sizes, such as 4 × 4 and 8 × 8. The strip wave block's geometric flow direction, which eliminates a considerable number of repeated sorting procedures. We use a similar optimization algorithm.

Two sort indexes are created:

- For each possible direction, the reordering index of the whole two-dimensional wavelet transform coefficient matrix is established, and the two-dimensional wavelet transform coefficient matrix is reordered into a one-dimensional vector
- The second index is set up to rearrange the wavelet coefficients of the one-dimensional vector after the one-dimensional wavelet transform is applied to each strip wave block

Then, the reordered one-dimensional vector is segmented (equivalent to the original two-dimensional matrix which is divided into blocks). The Lagrange function values in each direction are obtained. Finally, the direction of the minimum Lagrange function value corresponding to each vector segment is the best geometric flow direction of the corresponding block. The strip wave coefficients are obtained. Using this optimization, in the actual experiment, each martial arts image's feature extraction time (the size is 192 × 64 pixels) is 0.138 seconds. Compared with the original 1.4 seconds, the time consumption is significantly reduced. It is close to the HOG feature extraction time of each sample (0.12 seconds). The reduction of time consumption mainly depends on transforming a one-dimensional wavelet transform into a simple one-dimensional matrix. Then, the whole process only needs to implement a one-dimensional wavelet transform.

RETRACTED

## 5. Conclusion

A new method for the feature extraction and detection of martial arts is proposed based on the second-generation strip wave transform. To carry out learning information and recover the three-dimensional posture of martial arts in the image, statistical approaches in band wave transform as image descriptors are applied. Firstly, the optimization algorithm based on the original second-generation strip wave is used to improve the operation speed. Then, the relevant optimal parameters are established through experiments. Some statistical features are selected through the feature selection experiment and feature combination hoof. Finally, the maximum value of geometric flow is determined as an effective global feature representation. Different block sizes are used to reduce the dimension of features to further reduce the complexity of feature vectors. Then, the feature extraction method is used to extract the features of the training samples. The Gaussian process algorithm is used to train the predictor. The test image is tested on the database using the obtained predictor model. All the results are compared with feature extraction methods. From the results, it can be found that the maximum geometric flow feature can effectively represent the posture of martial arts. The image description ability of simple and basic motion sequences is better than that of the classical global image features. Different learning methods can obtain better tracking results and lower tracking errors. On the whole, from the test results of standard deviation, we can see that the tracking results of the data are relatively stable by using the maximum value feature of the strip wave. They have good adaptability and robustness in continuous image tracking, with slight fluctuation, which is more suitable for the description of martial arts images.

## Figures and Tables

**Figure 1:** Machine learning mode.

**Figure 2:** Performance comparison of different layers of the wavelet transform.

## Data Availability

The data used to support the findings of this study are included within the article.

## References

[1] Lili X., Yuan Z. (2020). Design and implementation of remote sensing monitoring system for resources and environment based on lidar technology. *J. Lasers*.

RETRACTED

[2] Chang L., Huixin Z., Qingqing P., Fanyi M. (2020). Design of high speed optical fiber video image transmission module based on embedded system. *Electron. Devices*.

[3] Hu Bin B. (2020). Design and application of automatic test system for optical transmission equipment. *Decision Exploration (middle)*.

[4] Hu H., Bo W. (2020). Design of 10 GB/s SFP+ optical module based on CWDM. *Communication Technology*.

[5] Shih T. T., Tseng P. H., Lai Y. Y., Cheng W. H. (2011). A 25 Gbit/s transmitter optical sub-assembly package employing cost-effective TO-CAN materials and processes. *Journal of Lightwave Technology*.

[6] Tian M. Q., Wang W., Song J. C., Song Y., Yan L., Xia Y. A dynamic load identification method for rock roadheaders based on wavelet packet and neural network.

[7] Geethalakshmi S., Narendran S., Ramalingam S., Pappa N. Optimization of fed-batch process for recombinant protein production in Escherichia coli using genetic algorithm.

[8] Tsai C. C., Tsai K. I., Su C. T. Cascaded fuzzy-PID control using PSO-EP algorithm for air source heat pumps.

[9] Takala T. M., Hirao Y., Morikawa H., Kawai T. Martial arts training in virtual reality with full-body tracking and physically simulated opponents.

[10] Banerjee A. K., Bhattacharyya G. K. (1979). Bayesian results for the inverse Gaussian distribution with an application. *Technometrics*.

[11] Yu Y., Liu B., Chen Z. (2018). Analyzing the performance of pseudo-random single photon counting ranging lidar. *Applied Optics*.

[12] Sokal N. O., Sokal A. D. (1975). Class E-A new class of high-efficiency tuned single-ended switching power amplifiers. *IEEE Journal of Solid-State Circuits*.

[13] Tang B. H., Zhou Z. X. The design of communication network optical fiber cable condition monitoring system based on distributed optical fiber sensor.

[14] Diethelm K., Ford N. J., Freed A. D. (2002). A predictor-corrector approach for the numerical solution of fractional differential equations. *Nonlinear Dynamics*.

[15] Zhao C. B., Wang M. J., Wang X. W. (2008). Self-optimization control in combustion system using genetic algorithms. *Coal Mine Machinery*.

[16] Zhang Y., Li Y., Liu Y., Yi G. (2020). Control of cricket system using LQR controller optimized by particle swarm optimization. *Journal of Physics: Conference Series*.

[17] Peng Z. PID control of temperature and humidity in granary based on improved genetic algorithm.

[18] Wu E., Koike H. Futurepose-mixed reality martial arts training using real-time 3d human pose forecasting with a rgb camera.

[19] Zhan L. M., Liu B., Fan L., Chen J., Wu X. M. Medical visual question answering via conditional reasoning.

[20] Xiao F., Liu B., Li R. (2020). Pedestrian object detection with fusion of visual attention mechanism and semantic computation. *Multimedia Tools and Applications*.

RETRACTED

[21] Zhang J., Liu Y., Liu H., Wang J. (2021). Learning local-global multiple correlation filters for robust visual tracking with k filter redetection. *Sensors*.

[22] Gu Y., Chen A., Zhang X., Fan C., Li K., Shen J. (2021). Deep learning based cell classification in imaging flow cytometer. *ASP Transactions on Pattern Recognition and Intelligent Systems*.

[23] Zhang J., Sun J., Wang J., Yue X. G. (2020). Visual object tracking based on residual network and cascaded correlation filters. *Journal of Ambient Intelligence and Humanized Computing*.

[24] Zhang J., Wang W., Lu C., Wang J., Sangaiah A. K. (2020). Lightweight deep network for traffic sign classification. *Annals of Telecommunications*.

[25] Liu R., Ning X., Cai W., Li G. (2021). Multiscale dense cross-attention mechanism with covariance pooling for hyperspectral image scene classification. *Mobile Information Systems*.

[26] Ding Y., Zhao X., Zhang Z., Cai W., Yang N. (2021). Multiscale graph sample and aggregate network with context-aware learning for hyperspectral image classification. *IEEE Journal of Selected Topics in Applied Earth Observations and Remote Sensing*.

[27] Cai W., Wei Z. (2020). Remote sensing image classification based on a cross-attention mechanism and graph convolution. *IEEE Geoscience and Remote Sensing Letters*.

[28] Huajie L. I., Wu J. (2011). The housing price forecasts of xia men based on BP neural network. *Journal of Shanxi Radio & TV University*.

[29] Li Y. Research on house price forecast based on grey system GM (1, 1).

[30] Wang Z., Zhang P., Sun W., Li D. (2021). Application of data dimension reduction method in high-dimensional data based on single-cell 3D genomic contact data. *ASP Transactions on Computers*.

[31] Sun W., Zhang P., Wang Z., Li D. (2021). Prediction of cardiovascular diseases based on machine learning. *ASP Transactions on Internet of Things*.

[32] Huang Z., Zhang P., Liu R., Li D. (2021). Immature apple detection method based on improved Yolov3. *ASP Transactions on Internet of Things*.

[33] Ning X., Gong K., Li W., Zhang L., Bai X., Tian S. (2020). Feature refinement and filter network for person re-identification. *IEEE Transactions on Circuits and Systems for Video Technology*.

[34] Ning X., Gou D., Dong X., Tian W., Yu L., Wang C. (2020). Conditional generative adversarial networks based on the principle of homologycontinuity for face aging. *Concurrency and Computation: Practice and Experience*.

[35] Zhang X., Yang Y., Li Z., Ning X., Qin Y., Cai W. (2021). An improved encoder-decoder network based on strip pool method applied to segmentation of farmland vacancy field. *Entropy*.

RETRACTED

[36] Fan M., Li Y. (2020). The application of computer graphics processing in visual communication design. *Journal of Intelligent and Fuzzy Systems*.

